# A Cohort Study of Rivaroxaban Combined with D-Dimer Dynamic Monitoring in the Prevention of Deep Venous Thrombosis after Knee Arthroplasty

**DOI:** 10.1155/2022/3965039

**Published:** 2022-04-19

**Authors:** Yongyong Dong, Guangbin Duan, Huihui Wang, Jia Ru, Yong Cui

**Affiliations:** Jincheng People's Hospital Orthopaedic Ward 1 Shanxi 048026, Orthopaedic Ward of Jincheng People's Hospital, No. 456 Wenchang East Street, Jincheng District, Shanxi Province, China

## Abstract

**Objective:**

To explore the cohort study of rivaroxaban combined with D-dimer dynamic monitoring in the prevention of deep venous thrombosis (DVT) after knee arthroplasty.

**Methods:**

Eighty-four patients with knee osteoarthritis who went through total knee arthroplasty from June 2019 to June 2021 in our hospital were arbitrarily assigned into the study group and the control group. The patients in the control group were cured with rivaroxaban anticoagulation after operation, and the study group was cured with dynamic monitoring of D-dimer on the basis of the control group. The incidence of postoperative DVT, pulmonary embolism (PE), and bleeding complications (incision ecchymosis and bleeding events) were compared. The related indexes such as drainage volume and blood transfusion volume were compared. The levels of activated partial prothrombin time (APPT), prothrombin time (PT), and D-dimer were dynamically monitored before and after operation. Visual analogue scale (VAS) was adopted to assess the degree of postoperative incision pain, the level of limb swelling before and after operation was measured, the circumference difference of affected limb was calculated, the ecchymosis area was assessed in the form of nine-palace grid, and the scores were compared.

**Results:**

According to the comparison of VAS score, there exhibited no remarkable difference before operation and on the first day after operation, but the VAS score decreased after operation, and the VAS score of the study group on the 3rd day, 7th day, and 14th day after operation was remarkably lower compared to the control group (*P* < 0.05). There exhibited no remarkable difference in drainage volume (*P* > 0.05), but the blood transfusion volume and total blood loss in the study group were remarkably lower (*P* < 0.05). There exhibited no remarkable difference in the level of PT on the 3rd day before operation and on the 3rd day after operation, but on the 7th day and 14th day after operation, the level of PT in the study group was remarkably higher (*P* < 0.05). The level of PT in the study group was remarkably higher (*P* < 0.05). There exhibited no remarkable difference in the level of APPT on the 3rd day before operation and on the 3rd day after operation, but on the 7th day and 14th day after operation, the level of APPT in the study group was remarkably higher (*P* < 0.05). The level of APPT in the study group was remarkably higher (*P* < 0.05). There exhibited no remarkable difference in the level of plasma D-dimer before operation (*P* > 0.05). The level of plasma D-dimer in the study group was lower (*P* < 0.05). In terms of the postoperative ecchymosis area score, the ecchymosis area score decreased remarkably after operation. Furthermore, the ecchymosis area score of the study group was remarkably lower (*P* < 0.05). In terms of the swelling degree of the affected limb, there exhibited no remarkable difference in thigh circumference and calf circumference before operation (*P* > 0.05), but after operation, the thigh circumference difference and calf circumference difference decreased, and the thigh circumference difference and calf circumference difference in the study group were lower (*P* < 0.05). The incidence of DVT in the study group was 16.67%, while that in the control group was 38.10%. No PE occurred in the two groups at the early stage after operation. There were 3 cases of incision ecchymosis, 1 case of bleeding event (incision oozing) in the study group, 11 cases of incisional ecchymosis, and 2 cases of bleeding event in the control group. In 3 patients with incisional bleeding, there were no obvious abnormalities in routine blood examination and blood coagulation indexes. The patients were given wound pressure bandaging and stopped using anticoagulants and changing wound dressings every day, all of which disappeared within 5 days. The incidence of early postoperative DVT and bleeding complications in the study group was lower (*P* < 0.05).

**Conclusion:**

Rivaroxaban combined with D-dimer dynamic monitoring has high clinical value in preventing DVT after knee arthroplasty and can effectively reduce the amount of blood loss during operation and the incidence of postoperative DVT, PE, and bleeding complications, which is worth popularizing to reduce the area of ecchymosis and the degree of pain after operation and shorten the recovery process.

## 1. Introduction

Deep venous thrombosis (DVT) of lower extremities is an acute nonbacterial inflammation induced by abnormal coagulation of blood in the deep veins of the lower extremities, blocking the deep veins of the lower extremities and resulting in blood flow disorders of the deep veins of the lower extremities [1]. DVT is a relatively common disease in Europe, the United States, and other countries. There are up to 580000 new DVT patients every year in the United States, and the annual prevalence rate of DVT in the United Kingdom is 0.01%. The number of deaths is much higher than that caused by tumors, AIDS, and traffic accidents.

As knee degenerative osteoarthritis is closely related to age factors, with the number of elderly people increasing year by year, the number of patients with knee degenerative osteoarthritis is also remarkably increased [2]. In China, the incidence of knee degenerative osteoarthritis in the middle-aged and elderly is as high as 60%-70%. For patients with moderate to severe knee osteoarthritis with significant pain, deformity, and knee dysfunction, total knee arthroplasty (TKA) is the mainstay of treatment for these conditions. Since TKA has obvious curative effect, effectively improving pain, deformity, and restoring activity function, it can remarkably enhance the quality of life of patients [3]. As a result, the number of patients undergoing knee replacements is increasing every year. The most common serious complications of TKA are DVT and PE [4]. Without anticoagulation, the incidence of DVT after TKA can be as high as 60%, and the incidence of fatal PE can be as high as 1.5% [5]. Drugs that can be used to prevent venous thromboembolism after TKA include warfarin, low molecular weight heparin, aspirin, oral factor Xa inhibitor, and direct thrombin inhibitors [6]. At present, low molecular weight heparin or factor Xa inhibitor is usually given for anticoagulation after TKA in China [7].

Rivaroxaban is a new type of oral anticoagulant, which directly inhibits factor Xa and thus plays an anticoagulant role [8–10]. D-dimer is a specific degradation product of fibrin hydrolyzed and cross-linked by plasmin, and it is one of the molecular markers of hypercoagulable state and secondary plasminogen hyperactivity in vivo [11–13]. The level of D-dimer usually begins to increase after operation and reaches the peak on the 7th day. If it remains at a high level on the 14th day after operation, the possibility of thrombosis should be considered [14, 15]. Based on this, 84 patients with knee osteoarthritis who underwent TKA in our hospital from June 2019 to June 2021 were studied as the object of our study, which is reported as follows.

## 2. Patients and Methods

### 2.1. Participant Information

84 cases with osteoarthritis of the knee admitted to our hospital from June 2019 to June 2021 were randomly divided into a study group and a control group. The patients in the control group were cured with rivaroxaban anticoagulation after operation, and the study group was cured with dynamic monitoring of D-dimer on the basis of the control group. In the control group, the age was 55-70 years old, with an average of 63.23 ± 6.17 years, including 23 males and 18 females, while in the study group, the age was 54-71 years old, with an average of 64.58 ± 5.46 years, including 19 males and 17 females. There exhibited no statistical significance in the general data. This study was permitted by the Medical Ethics Association of our hospital, and all patients noticed informed consent.

The inclusion criteria were as follows: (1) patients who underwent unilateral total knee arthroplasty due to knee osteoarthritis; (2) patients without cognitive, language, and intellectual impairment and patients with basic reading and writing ability; (3) no preoperative venous thrombotic disease or history; (4) good compliance and real-time follow-up; (5) there were no serious medical diseases, such as heart, liver, kidney functional injury or failure.

Exclusion criteria are as follows: (1) patients with severe heart, liver, renal insufficiency, malignant tumors, and other diseases; (2) patients with sensitive constitution or allergic to a variety of drugs (traditional Chinese medicine or western medicine); (3) patients unwilling to use tested drugs; (4) patients with bleeding tendency or accompanied with coagulation dysfunction; (5) pregnant women and lactating patients; (6) patients who could not comply with treatment and late rehabilitation physiotherapy because of mental and psychological diseases.

### 2.2. Treatment Methods

#### 2.2.1. Preoperative Preparation

All patients were examined routinely before operation, such as blood, urine routine, liver and renal function, electrolyte, coagulation, blood glucose, heart and lower limb arteriovenous Doppler ultrasonography, and other related examinations, to understand the overall condition of the patient, the venous valvular function of the lower extremities, and the patency of the arteries and veins of the lower extremities, to correct the preoperative examination index within the safe range, to avoid the occurrence of perioperative complications, and especially to reduce the risk of infection and DVT as much as possible. Preoperative health education was carried out by medical staff to make patients understand the principle and adverse factors of DVT formation, to make patients understand the necessity of early joint exercise after operation, and to guide them to learn the methods of exercise. It is suggested that patients should improve their lifestyle, such as abandoning tobacco, alcohol, and other adverse factors, healthy diet, and so on.

#### 2.2.2. Operation Method

All the patients underwent total knee arthroplasty, and the operation was performed by the same group of doctors in our department. All patients were anesthetized with combined spinal-epidural anesthesia. All the surgical approaches were performed with a median longitudinal incision of the knee joint, and the length of the incision was about 15 cm.

The procedure should minimize the extent of incisions and dissections and the correct use of tourniquets (position, timing, and pressure strictly in accordance with standards) to avoid unnecessary vascular damage. Complete intraoperative haemostasis and appropriate fluid replacement to avoid dehydration. Reduce blood viscosity and, if necessary, transfuse blood to replenish circulating blood volume. The surgical incision is closed in layers carefully and the drainage tube is placed into the other incision and wrapped with a sterile cotton pad.

#### 2.2.3. Postoperative Treatment

Control group: all patients in this group were given rivaroxaban (approval number: H20090207, enterprise name: Bayer Pharma AG) once a day, each time 10 mg oral administration; the course of treatment was 15 days, that was, from the 1st day to the 15th day after operation. The study group: on the basis of the control group, the dynamic monitoring of D-dimer was combined, and the corresponding prevention and treatment measures were taken in time according to the dynamic monitoring results. All the patients were given the same basic prevention and physical prevention, and routine pain relief, infection prevention, knee functional exercise, nursing, and rehabilitation treatment were carried out at the same time, so as to avoid or reduce the occurrence of perioperative adverse events as far as possible, so as to create conditions conducive to the recovery of postoperative patients. For example, patients were warned to abandon tobacco and alcohol, light, and balanced diet and adopt a healthy lifestyle before operation; the same drug treatment was used after TKA, such as infection prevention, pain relief, and swelling reduction; after operation, ice bags wrapped in soft towels were placed around the affected knee joint and cold compress the incision to facilitate swelling reduction and analgesia; after operation, the affected limb was immediately bandaged with elastic straps from the dorsum of the foot to the knee joint. After the operation, the affected limb was padded high to facilitate reflux and detumescence, with a height of 15-20 cm, slightly above the level of the heart; when the postoperative anesthetic effect disappears, guide the patient to carry out functional exercise on the bed, such as active extension of the ankle joint and relaxation and contraction of the quadriceps femoris and gastrocnemius, guide the patient's family members to give the affected limb proper massage, and help the patient carry out functional exercise. 2-3 days after operation, the negative pressure drainage tube was removed, and the affected limb was used for lower limb functional exercise with CPM machine.

### 2.3. Observation Index

#### 2.3.1. Clinical Data Collection Table

Self-designed, including four parts, the first part mainly includes the patient's name, sex, age, past disease history, and other basic information. The second part is the preoperative situation: preoperative fasting time, preoperative PT, APPT, and D-dimer levels. The third part is the intraoperative indicators: drainage, blood transfusion, and total blood loss. The fourth part is the postoperative recovery indicators: the incidence of postoperative venous thrombosis, PE, and bleeding complications, statistics of the degree of swelling of patients in the group, and so on.

#### 2.3.2. VAS Scoring

VAS [16]: 0: painless; <3: mild pain, bearable; 4-6: pain and affects sleep; 7-10: strong pain, unbearable, affecting life.

#### 2.3.3. Biochemical Index

Biochemical examination was carried out by automatic biochemical analyzer. PT, APPT, and the level of D-dimer were calculated in the two groups.

#### 2.3.4. Ecchymosis Area

The area of ecchymosis was measured in the form of nine-palace grid, and the area of each grid was 1 cm^2^. The postoperative ecchymosis area of the two groups was recorded, and the score was calculated. The scoring criteria were 0: no obvious ecchymosis, 1: ecchymosis area <3 cm^2^, 2: ecchymosis area 3-12 cm^2^, and 3: ecchymosis area >12 cm^2^.

#### 2.3.5. Diagnosis of Symptomatic VTE

Four items of coagulation + D-dimer examination and bilateral deep vein ultrasonography of lower extremities except lower limb DVT were performed in all patients who underwent TAK operation. On the third day after operation, bilateral deep vein ultrasonography and coagulation + D-dimer examination were performed to determine whether DVT occurred after TKA. The diagnostic criteria were as follows: (1) the venous lumen could not be closed; (2) the venous lumen was hypoechoic or anechoic; (3) pulsed Doppler ultrasound showed that there was no blood flow or the frequency spectrum did not change with respiration; (4) there was no blood flow signal or only a small amount of blood flow signal was detected in the thrombotic vein. If the patient had chest tightness and chest pain after operation (except precordial pain), consult a physician. According to the consultation opinion, chest enhancement CT or pulmonary angiography should be performed to determine whether the patient had PE.

### 2.4. Statistical Analysis

The measurement data were subjected to normal distribution and chi-square analysis prior to statistical analysis to satisfy the requirement of normal or approximately normal distribution, expressed as ±*s*. Repeated measurement data were subjected to ANOVA. The two groups were compared using the *t*-test, and the count data were expressed as *n* (%) by the *χ*^2^ test. SPSS21. 0 statistical software was used. The differences exhibited statistically remarkable (*P* < 0.05).

## 3. Results

### 3.1. VAS Score Comparison

There exhibited no remarkable difference in VAS scores before operation and on the first day after operation, but the VAS scores decreased after operation, and the VAS scores of the study group on the 3rd day, 7th day, and 14th day after operation were remarkably lower compared to the control group (*P* < 0.01). All the detailed results are indicated in Table 1.

### 3.2. Comparison of Related Indexes Such as Drainage Volume, Blood Transfusion Volume, and Recessive Blood Loss

There exhibited no remarkable difference in drainage volume (*P* > 0.05), but the blood transfusion volume and total blood loss in the study group were remarkably lower (*P* < 0.05). The results are shown in Table 2.

### 3.3. Comparison of PT between Two Groups

There exhibited no remarkable difference in the level of PT before operation and on the 3rd day after operation. But on the 7th day and 14th day after operation, the level of PT in the study group was remarkably higher (*P* < 0.05). All the detailed results are indicated in Table 3.

### 3.4. Comparison of APPT between Two Groups

There exhibited no remarkable difference in the level of APPT before and 3 days after operation. But on the 7th day and 14th day after operation, the level of APPT in the study group was remarkably higher (*P* < 0.05). All the detailed results are indicated in Table 4.

### 3.5. Comparison of Plasma D-Dimer Levels between Two Groups

There exhibited no remarkable difference in the level of plasma D-dimer before operation (*P* > 0.05). The level of plasma D-dimer in the study group was remarkably lower (*P* < 0.05). All the detailed results are indicated in Table 5.

### 3.6. Comparison of Postoperative Ecchymosis Area Score

In terms of the postoperative ecchymosis area score, the two groups decreased remarkably after operation. Compared with the control group, the ecchymosis area score of the study group was remarkably lower (*P* < 0.05). All the detailed results are indicated in Figure 1.

### 3.7. Comparison of Swelling Degree of Affected Limb

In terms of the swelling degree of the affected limb, there exhibited no remarkable difference in thigh circumference and calf circumference before operation (*P* > 0.05). The difference in thigh circumference and calf circumference in the study group was remarkably lower (*P* < 0.05). All the detailed results are indicated in Table 6.

### 3.8. Comparison of Early Postoperative DVT, PE, and Bleeding Complications

There exhibited no remarkable difference in the incidence of DVT on the 3rd day. The incidence of DVT in the study group was 16.67%, while that in the control group was 38.10%. No PE occurred at the early stage after operation. There were 3 cases of incision ecchymosis, 1 case of bleeding event (incision oozing) in the study group, 11 cases of incisional ecchymosis, and 2 cases of bleeding event (incision oozing) in the control group. Among 3 patients with incisional bleeding, there were no obvious abnormalities in routine blood examination and blood coagulation indexes. The patients were given wound pressure bandaging, stopped using anticoagulants, and changing wound dressings every day, all of which disappeared within 5 days. The incidence of early postoperative DVT and bleeding complications (incision ecchymosis and bleeding events) in the study group were remarkably lower compared to the control group (*P* < 0.05). All the detailed results are indicated in Figure 2.

## 4. Discussion

DVT of lower extremities is an acute nonbacterial inflammation induced by abnormal coagulation of blood in the lumen of deep veins of lower extremities, blocking the deep veins of lower extremities and causing blood flow disorders of deep veins of lower extremities [17–19]. The number of DVT-related deaths is much higher than that derived from tumors, AIDS, and traffic accidents [17]. The investigation indicates that the detection rate of DVT is as high as 20.7% and shows a growing trend. As knee degenerative osteoarthritis is closely related to age factors, with the number of elderly people in China increasing year by year, the number of patients with knee degenerative osteoarthritis also increased remarkably [20, 21]. Considering that TKA has remarkable curative effect, effectively improve pain, deformity, and restore activity function, it can remarkably improve the quality of life of patients. Therefore, the number of patients undergoing TKA is increasing year by year, but the most common serious complication of TKA is DVT. How to prevent and treat DVT safely and effectively and improve the efficacy of surgery and patients' quality of life and other research has become an important medical task and urgent practical needs.

Rivaroxaban is a new generation of representative oral antithrombotic agents. This kind of drug does not need antithrombin during anticoagulation; it directly binds to the active site of factor Xa and has high affinity, thus inhibiting the activity of factor Xa [22–25]. Given that rivaroxaban can highly competitively inhibit this factor, and it is located at the core of endogenous and exogenous coagulation pathways, which can effectively block the coagulation process, prolong PT and APPT, effectively anticoagulated, and inhibit thrombosis [23], a number of clinical trials have indicated that rivaroxaban is effective in the prevention and treatment of venous thrombosis. Compared with the most commonly used low molecular weight heparin drugs, rivaroxaban has the following remarkable advantages [26–28]: (1) easy to use and high degree of patient compliance; the drug is taken once a day, one tablet at a time, do not need to regularly monitor blood coagulation function, and adjust the dose, convenient for out-of-hospital use; (2) less pain: there was no injection pain and no discomfort such as itching at the injection site; (3) the individual difference was small; the drug is not disturbed by individual factors, such as age, sex, and body mass, and the treatment window is wider; (4) it is safer; without the function of antiplatelet aggregation, the risk of bleeding is lower; (5) the bioavailability is high and the performance is stable. Oral administration of the drug has 80% bioavailability, and 10 mg/d can achieve the effect of preventing thrombus.

D-dimer is a specific degradation product of cross-linked fibrin formed by activation of fibrinogen and then hydrolyzed by plasmin. D-dimer is the simplest degradation product of fibrin, which was mainly from cross-linked fibrin clot dissolved by plasmin. Its concentration can change with trauma, surgery, pregnancy, and thrombosis, thus reflecting the anticoagulation system and fibrinolysis system of the human body. Some studies have indicated that D-dimer can be adopted in the diagnosis of lower extremity DVT and PE [29]. Some reports have indicated that the abnormal increase of D-dimer is positively correlated with the probability and size of thrombosis [30]. However, some scholars have proved that the specificity of D-dimer in predicting human thrombosis is poor, which may be due to the influence of trauma, release of inflammatory factors, bleeding, and complications. The D-dimer in most patients is remarkably higher compared to the normal value [31]. In this current study, 84 patients who underwent TKA were enrolled. The results indicated that the VAS scores of the two groups decreased after operation. The VAS scores of the study group on the 3rd, 7th, and 14th day after operation were remarkably lower compared to that in the control group. The blood transfusion volume and total blood loss in the study group were remarkably lower. On the 7th day and 14th day after operation, the levels of PT and APPT in the two groups increased, and the levels of PT and APPT in the study group were remarkably higher. On the 3rd day after operation, the plasma D-dimer increased remarkably and decreased on the 7th and 14th day after operation. Moreover, the level of D-dimer in the study group was lower. In terms of the postoperative ecchymosis area score, the ecchymosis area score decreased remarkably, the ecchymosis area score of the study group was remarkably lower, and the thigh circumference difference and calf circumference difference of the study group were lower. In addition, the incidence of DVT was 16.67% in the study group and 38.10% in the control group. No PE occurred at the early stage after operation. There were 3 cases of incision ecchymosis, 1 case of bleeding event (incision oozing) in the study group, 11 cases of incisional ecchymosis, and 2 cases of bleeding event (incision oozing) in the control group. In 3 patients with incisional bleeding, there were no obvious abnormalities in routine blood examination and blood coagulation indexes. The patients were given wound pressure bandaging, stopped using anticoagulants, and changed wound dressings every day, all of which disappeared within 5 days. The incidence of early postoperative DVT and bleeding complications (incision ecchymosis and bleeding events) in the study group was lower.

In conclusion, rivaroxaban combined with D-dimer dynamic monitoring has high clinical value in preventing DVT after knee arthroplasty and can effectively reduce the amount of blood loss during operation and the incidence of postoperative DVT, PE, and bleeding complications, which is worth popularizing to reduce the area of ecchymosis and the degree of pain after operation and shorten the recovery process.

## Figures and Tables

**Figure 1:** Comparison of postoperative ecchymosis area integral scores between two groups [$\bar{x}\pm s$, points] of patients after operation. The black bar represents control group, and the grey bar represents research group.

**Figure 2:** Comparison of early postoperative complications of deep vein thrombosis, pulmonary embolism, and hemorrhage between two groups [*n*/%].

**Table 1:** Comparison of VAS scores between the two groups [$\bar{x}\pm s$, points].

Group	Cases	Before operation	The first day after operation	The third day after operation	The seven days after operation	The fourteen days after operation
Control group	42	9.08 ± 2.14	8.53 ± 0.76	5.56 ± 1.09	3.54 ± 0.47	1.87 ± 0.72
Research group	42	8.98 ± 2.03	8.34 ± 0.41	5.11 ± 0.76	2.13 ± 0.04	1.03 ± 0.76
*t*		0.220	1.426	2.195	19.372	5.200
*P*		0.827	0.158	0.031	<0.01	<0.01

**Table 2:** Comparison of drainage volume, blood transfusion volume, and recessive blood loss between the two groups [$\bar{x}\pm s$].

Group	Cases	Drainage volume (mL)	Blood transfusion volume (mL)	Total blood loss (mL)
Control group	42	64.02 ± 63.45	20.08 ± 11.24	1096.31 ± 195.46
Research group	42	64.12 ± 70.13	8.35 ± 6.21	894.24 ± 188.53
*t*		0.007	5.920	4.822
*P*		0.995	<0.01	<0.01

**Table 3:** Comparison of PT between the two groups before and after treatment [$\bar{x}\pm s$, s].

Group	Cases	Before operation	Third days after operation	Seven days after operation	Fourteen days after operation
Control group	42	11.52 ± 11.14	10.74 ± 1.02	12.34 ± 1.29	12.43 ± 1.07
Research group	42	11.63 ± 1.28	11.06 ± 1.33	13.01 ± 1.56	13.11 ± 1.66
*t*		0.064	1.237	2.145	2.231
*P*		0.950	0.220	0.035	0.028

**Table 4:** Comparison of APPT between the two groups before and after treatment [$\bar{x}\pm s$, s].

Group	Cases	Before operation	Third days after operation	Seven days after operation	Fourteen days after operation
Control group	42	35.08 ± 4.87	34.15 ± 4.67	36.17 ± 4.15	36.36 ± 4.08
Research group	42	35.34 ± 5.07	35.02 ± 3.73	38.41 ± 4.38	38.53 ± 4.52
*t*		0.240	0.943	2.406	2.310
*P*		0.811	348	0.018	0.023

**Table 5:** Comparison of plasma D-dimer between the two groups [$\bar{x}\pm s$, mg/L].

Group	Cases	Before operation	Third days after operation	Seven days after operation	Fourteen days after operation
Control group	42	1.45 ± 0.34	2.35 ± 0.42	1.59 ± 0.23	1.18 ± 0.42
Research group	42	1.48 ± 0.46	2.11 ± 0.56	1.38 ± 0.51	0.93 ± 0.31
*t*		0.340	2.222	2.433	3.104
*P*		0.735	0.029	0.017	0.003

**Table 6:** Comparison of the swelling degree of the affected limb between the two groups [$\bar{x}\pm s$].

Group	*N*	Thigh circumference difference (example)		Leg circumference difference (example)	
		Before operation	Fourteen days after operation	Before operation	Fourteen days after operation
Control group	42	15.47 ± 4.68	13.98 ± 2.23^a^	16.55 ± 3.67	14.43 ± 4.57^a^
Research group	42	15.93 ± 4.41	11.54 ± 2.71^b^	16.43 ± 3.78	10.94 ± 1.36^b^
*t*		0.464	4.506	0.148	4.744
*P*		0.644	<0.01	0.883	<0.01

Note: the control group before and after nursing; ^a^*P* < 0.05; the study group before and after nursing; ^b^*P* < 0.05.

## Data Availability

No data were used to support this study.
